# Effect of Acupressure on Health-Related Quality of Life in Patients with Polycystic Ovarian Syndrome: A Randomized Clinical Trial

**DOI:** 10.1155/2022/2920132

**Published:** 2022-06-06

**Authors:** Marzieh Nekooi, Fatemeh Bazarganipour, Mohammad Zoladl, Reza Heshmat, Shahintaj Aramesh, Nazafarin Hosseini

**Affiliations:** ^1^Student Research Committee, Yasuj University of Medical Sciences, Yasuj, Iran; ^2^Social Determinants of Health Research Center, Yasuj University of Medical Sciences, Yasuj, Iran; ^3^Shahid Beheshti University of Medical Sciences, Tehran, Iran; ^4^Acupuncture Medicine Association, Tehran, Iran; ^5^Department of Gynecology and Obstetrics, Yasuj University of Medical Sciences, Yasuj, Iran

## Abstract

The present study was conducted to determine the effect of acupressure on health-related quality of life in patients with polycystic ovary syndrome. This study was a double-blind, randomized clinical trial with a control group. Ninety-six patients with polycystic ovary syndrome from Mofateh gynecological clinic in Yasuj in Iran were enrolled according to the inclusion criteria. Patients were randomly assigned to intervention and control groups. In the intervention group, pressure on the points, Ren3, Ren4, Liv3, Sp6, and Sp10 and in the control group, pressure on sham points were performed for 6 weeks (2 sessions per week). The primary outcome was health-related quality of life, measured by the modified polycystic ovary syndrome health-related quality of life questionnaire (MPCOSQ). The secondary outcomes were total testosterone levels and clinical symptoms in patients with polycystic ovary syndrome. The outcome variables were measured before the intervention at week 0 (baseline) and after the intervention at week 18 (12 weeks after the end of intervention). The results indicated that at week 18, the score of clinical symptoms and the total testosterone level of the intervention group were lower than those of the control group. The health-related quality of life score in the intervention group was higher than that in the control group, which was statistically significant (*P* < 0/05). Therefore, acupressure in these points is recommended as a practical and effective method of treating polycystic ovarian syndrome.

## 1. Introduction

Polycystic ovarian syndrome (PCOS) is one of the most common clinical endocrine disorders of the reproductive system in women of childbearing age [1, 2]. The prevalence of this syndrome globally is 5–15% [3], and in Iran, based on the Rotterdam criterion, it is 14.6% [4]. The metabolic risk factor for PCOS is typically an increase in testosterone levels due to a decrease in sex hormone-binding globulin (SHBG). These people have higher levels of luteinizing hormone (LH), follicle-stimulating hormone (FSH), adrenocorticotrophic hormone (ACTH), insulin, cholesterol, and triglycerides compared to healthy people [5]. These changes cause ovulation disorders, menstrual irregularities, and infertility, resulting in reduced health-related quality of life (HRQOL) [6]. In addition, these changes cause physical manifestations such as changes in appearance and especially obesity, hirsutism, acne, hair loss, behavioural changes, and sexual orientation changes that can affect the female identity and thus the HRQOL [7, 8]. Health-related quality of life, satisfaction, and happiness affect a person's health and are a multidimensional concept that includes physical, mental, cultural, and social dimensions [9]. In a qualitative study in Iran, the domains of HRQOL of patients with PCOS have emerged in six domains of emotional disturbance, hirsutism, infertility, weight, menstruation, and acne disorders [10].

Due to the lack of definitive treatment for PCOS, disease management should improve the health-related quality of life by improving symptoms and preventing long-term complications of the disease [11]. Complementary and alternative therapies are harmless therapies that do not seem to have negative consequences [12]. Acupressure is based on the theory of meridians and believes that vital energy (qi) is distributed throughout the body by meridians and the imbalance of vital energy flow leads to disease or pain [13]. In traditional Chinese medicine, PCOS combines amenorrhea, irregular menstruation, and infertility. The most involved organs are the kidneys, liver, and spleen. PCOS is mainly caused by the following reasons: (1) yang deficiency due to obstruction of Yang and Ren canals that causes poor blood flow to the uterus and amenorrhea. (2) Lack of splenic Qi causes fluid storage in the body and turns it into sputum and moisture, which blocks the Ren and Yang canals and blocks Qi of blood flow and causes amenorrhea. (3) Obstruction of Chang and Ren canals due to liver Qi stagnation and blood stasis causes amenorrhea [14].

Acupressure and acupuncture activate sensory nerve fibbers by stimulating receptors in skeletal muscles. These signals are transmitted to the spinal cord through spinal reflexes and may modulate a sympathetic output to target organs in the same area of the nerve. It similarly and effectively treats PCOS by affecting the hypothalamic-pituitary-ovarian axis and increasing central beta-endorphin [15]. 14 meridians in the body are used in acupuncture and acupressure [16]. Acupressure is the pressure on and stimulation of these points that improve or increase the flow of energy and can ultimately lead to the improvement of the disease [17]. The main points selected are the renal meridians, and several points of acupressure related to the hepatic and splenic canal affecting PCOS can be used [18].

In a study, Ling et al. revealed the effect of acupuncture on improving the quality of life of patients with depression [19]. By studying the effect of acupuncture on patients with polycystic ovaries, Lim et al. found a significant reduction in the interval between menstruation and follicle-stimulating hormone levels, the ratio of luteinizing hormone to follicle-stimulating hormone, progesterone, and free androgen index (FAI) [20].

A study about the effect of acupressure on the HRQOL of these patients has not been found yet by researchers. Therefore, due to the patients' low health-related quality of life, this study was conducted to determine the effect of acupressure on the health-related quality of life of patients with polycystic ovarian syndrome. The other purpose of this study was to determine the effect of acupressure on the testosterone levels and clinical symptoms of the patients.

## 2. Materials and Methods

### 2.1. Study Design

This randomized clinical trial was registered on the Iranian Registry of Clinical Trials Website (IRCT); ID: IRCT20180725040587N1. The intervention was performed from July 2018 to November 2018. The primary outcome was health-related quality of life in patients with polycystic ovary syndrome (PCOS). The secondary outcomes were total testosterone levels and clinical symptoms in the patients. In this study, control and intervention groups participated. Before and after the intervention, the outcomes were compared between the two groups, within the groups, at week 0 (baseline), and week 18 (12 weeks after the end of intervention) [21]. The intervention was double-blind. Patients and statistical analysts did not know in which group they were.

### 2.2. Participants and Sampling

The participants consisted of patients with polycystic PCOS ovary syndrome referred to Mofateh gynecological clinic in Yasuj, Iran, who were eligible, and met the inclusion criteria.

Inclusion criteria were as follows: PCOS approved by the gynecologist, married, obtaining a minimum baseline score (1.3 points of the MPCOSQ), health-related quality of life questionnaire, absence of male infertility factor (confirmed by spermogram test), age 15–45 years [22], and history of infertility approved by a gynecologist and approving PCOS according to the Rotterdam standard. The Rotterdam diagnostic criteria include the following: (1) polycystic ovaries visualized on an ultrasound scan (presence of 12 follicles or more in one or both ovaries and/or increased ovarian volume, i.e., >10 ml), (2) clinical signs of hyperandrogenism (hirsutism score based on hirsutism score greater than 7 or obvious acne) and/or elevated plasma testosterone (testosterone >2.0 nmol/l), and (3) having an interval between menstrual periods >35 days and/or amenorrhea, defined as the absence of vaginal bleeding for at least 6 months (i.e., 199 days) [23].

Exclusion criteria were as follows: Any systemic or endocrine and neurological disease based on the patient's declaration (confirmed by a specialist), addiction, use of any hormonal drugs except clomiphene, discontinuation of clomiphene, and lack of cooperation of the participants to continue treatment.

In the present study, in order to estimate the sample size, the mean standard deviation of the six areas of quality of life-related measurement of patients with PCOS, Bazarganipour et al. study was used. Based on the type 1 error = 0.05 (95% confidence level), the type 2 error = 20% (power 80%) and effect size = 1, and *σ* = 1.59, the number of participants in each group was estimated to be 39.64 [22] using the following formula:

(1) $$\begin{array}{c} n=\frac{2*{\left(\text{Z}1-\left(\alpha /2\right)+\text{Z}1-\beta \right)}^{2}*\sigma^{2}}{d^{2}}. \end{array}$$

The sample size was calculated considering 20% of possible participants drop. Finally, 96 participants were included in the study as a sample. Forty-eight people were assigned to each group.

The patients who participated in the present study were selected by the convenience sampling method. They were randomly assigned to the intervention and control groups in a randomized block method using sample randomizer software.

### 2.3. Instruments and Data Gathering

Data were collected through a demographic and fertility information questionnaire, a checklist of clinical symptoms, and a modified polycystic ovary syndrome health-related quality-of-life questionnaire (MPCOSQ), at week 0 (baseline), and week 18 (12 weeks after intervention) [21].

- Demographic and fertility information questionnaire includes age, body mass index (BMI), duration and type of infertility, number of children, ethnicity, level of education, and employment status.
- Checklist of clinical symptoms and laboratory signs:
- Clinical symptoms: Clinical symptoms, including hirsutism, acne, alopecia, and menstrual problems, were recorded in a checklist by the researcher (community health nurse) based on the following indicators and investigation by the researcher and asking the patients.
- Hirsutism was measured and scored by the Freeman Galloy scale. A score of 8 or higher was the criterion for hirsutism. The latest hirsutism scoring system is the Freeman Galloway Scale, a suitable tool for the clinical examination of hirsutism. This scale was first proposed by Hatch et al. and adjusted by Freeman and Galloy and was limited to nine androgen-sensitive areas, including lips, chin, front of chest, abdomen, pubis, arm, inner thigh, back, and buttocks. The score of hirsutism is obtained from the sum of nine points of the body, for which a score of 8 or more is the criterion of hirsutism [24].
- The Global Acne Grading System was used to assess acne. This scale considers six parts of the face, chest, and upper back based on the level of involvement, distribution, and density of the pilosebaceous units. The border of the face was determined by the growth path of hair, chin, and ears. Each of the six parts was scored on a zero-to-four scale, with the most severe injury in each part determining that area's score. Then, the score of each part was multiplied by the factor score. The factor score varies based on the area involved, as follows.
- Forehead: 2, right or left cheek: 2, nose: 1, chin: 1, and chest and upper back: 3; therefore, the total acne score is the multiplication of the factor score and total score of the affected areas [25].
- Based on the Ludwig scale of female hair loss, alopecia is defined as a moderate and severe reduction in the hair density on the scalp and hair loss on the forehead and temples [26].
- Menstrual status was defined as follows.
- Regular menstruation: The interval between two periods is 21–35 days.
- Irregular menstruation: The interval between two periods is less than 35 days.
- Oligomenorrhea: The interval between two periods is more than 35 days,
- Amenorrhea: Menstrual symptoms interval of more than six months [22].
- Laboratory signs include total testosterone levels, in which patients were referred to the laboratory before the intervention (week 0) and week 18 (12 weeks after the intervention) in the morning of fasting. To determine total testosterone levels, a blood sample (5 cc) was taken from each participant to extract a serum sample. Total testosterone levels of the participants were measured using a monobond kit and ELISA method by a Human device made in Germany. Device calibration was also considered. The researcher collected the results from the laboratory and recorded in a checklist of clinical and laboratory symptoms.
- Modified polycystic ovary syndrome health-related quality of life questionnaire (MPCOSQ) included 30 questions about 6 domains of health-related quality of life: emotional disturbance (8 items), hirsutism (5 items), infertility (4 items), weight (5 items), menstrual (4 items), and acne (4 items). A seven-point Likert scale was used to score, in which a score of 7 means no problem and a score of 1 means a disorder in quality of life [10, 27]. The validity and reliability of the MPCOSQ in the Iranian population have been confirmed by Bazarganipour et al. [22].

The Echo Doctor electroacupuncture machine, model LY-508B, made in China and under the British license, was used to find the acupressure points. The machine had a frequency of 23 Hz. Hearing the beep and changing the number on the digital screen, acupressure points were determined.

### 2.4. Intervention

Acupressure intervention was performed by a researcher (community health nurse) with an acupressure certificate. The main points were selected from the renal meridians, and several points of acupressure related to the hepatic and splenic canals affecting PCOS were used [18]. The Echo Doctor electroacupuncture machine was used to find the acupressure points.

Patients lay on the bed and relaxed completely to receive acupressure in the intervention group. Acupressure intervention was performed on the pressure points of Ren-3, Ren-4, Liv3, Sp10, and Sp6. The intervention was performed twice a week for 6 weeks [28]. The third point of the liver (Liv3) is located between the first and second metatarsal bones of the sole, at a distance of four cuns from the toe. The sham point of the Liv3 is located between the third and the fourth toes, which are not in the meridian line [29] (Figure 1(a)).

The sixth point of the spleen (SP6) is located at a distance of four cuns above the inner ankle of the foot and the posterior edge of the tibia. The sham point of the SP6 was considered to be about one centimetre outside the SP6, which is not in the meridian line (Figure 1(b)). The tenth point of the spleen (SP10) is five cuns away from the upper inner part of the patellar edge of the knee in a curved position. The sham point of the SP10 was considered to be about one centimetre lower than the SP10, which is not in the meridian line (Figure 1(c)).

The Ren-3 point is in the midline of the abdomen, 4 cuns below the umbilicus, and 1 cun above the symphysis pubis. The Ren-4 point is located in the midline of the abdomen, three cuns below the umbilicus, and one cun above the symphysis pubis [20]. The sham points of Ren-3 and Ren-4 points were considered to be about one centimetre outside from real acupoints, which are not in the meridian line (Figure 1(d)).

In the control group, interventions were performed similarly to the intervention group. The only difference was that the pressure was performed on the false or sham points in one to two centimetres near the main point.

Acupressure points and sham points were determined by a laser point detector. In this way, when the device was in the path of the acupressure point, it started to sound the alarm (this sound was due to the potential difference between the acupressure points and other points). In the intervention, the pressure was performed circularly by counting from 1 to 6, there was a break with counting from 1 to 2. It was performed at each point for five minutes with the amount of pressure to the extent that the point under pressure becomes numb or tingling. In both intervention and control groups, three sessions of intervention were performed by the researcher and the patient was trained during the intervention. The patient conducted three sessions of intervention in the clinic and under the researcher's supervision. Another six sessions of acupressure or pressure on false points were assigned to the patient at home. The intervention group was given information about acupressure points and how to use pressure. Pamphlets and videos about false pressure points and how to apply pressure were given to the control group and they were asked to register for sessions in the forms provided to them. It should be noted that all patients taking clomiphene at a dose of 50 mg per day from the third day of the menstrual period to the ninth day were treated routinely. The measurement periods of the research variables were baseline (week 0) and week 12 after the intervention (week 18) [21].

### 2.5. Ethical Considerations

This study was approved by the Research Ethics Committee (REC) of Yasuj University of Medical Sciences (YUMS) with ID code: IRYUMS.REC.1397.035. Written informed consent was obtained from all patients to participate in the study and they were allowed to leave the study voluntarily. Other ethical considerations were maintaining their privacy and confidentiality of the information, maintaining the temperature, light, and proper ventilation of the room, and not imposing any costs on patients to participate in the study. At the end of the study, the control group was given the necessary training on acupressure intervention.

### 2.6. Data Analysis

SPSS software version 21 was used to analyze data in this study. Data were analyzed by considering the data from the natural distribution based on the central limit theorem concerning the presence of 48 people in each study group. Independent *t*-test, Chi-square test, and independent *t*-test were used for analyzing data.

## 3. Results

Ninety-six patients with PCOS participated in the study. Forty-eight patients were in the acupressure intervention group, and the other forty-eight patients were in the control group. All participants remained until the end of the study (Figure 2).

The mean age of study participants was 32.7 ± 3.1 years, and their body mass index was 26.5 ± 2.1. At the beginning of the study, there was no statistically significant difference between the groups regarding age, occupation, education, body mass index (BMI), duration of infertility, number of children, menstrual status, and type of infertility (*P* > 0.05) (Table 1).

There was no statistically significant difference between the studied groups in terms of clinical symptoms (acne, hirsutism, and alopecia) and total testosterone levels at baseline (*P* > 0.05), but a significant decrease in the mean of these variables was shown in the intervention group compared to the control group after the intervention (*P* < 0.05) (Table 2).

In the intervention group, the mean scores in clinical symptoms (acne, hirsutism, and alopecia) and total testosterone levels after the research intervention compared to the basal point of the study decreased significantly (*P* < 0.05). However, in the control group, the mean scores on clinical symptoms (acne, hirsutism, and alopecia) and total testosterone levels at the baseline of the study compared to after the research intervention did not show a statistically significant difference (*P* > 0.05) (Table 3).

Before the intervention, there was no significant difference between the control and intervention groups in the mean score of health-related quality of life and its domains, including emotional disturbance, weight, infertility, menstrual, hirsutism, and acne, but after the intervention, a significant improvement in the mean score of these variables was shown in the intervention group compared to the control group (*P* < 0.05) (Table 2). The mean score of health-related quality of life and its areas including emotional disturbance, weight, infertility, menstrual, hirsutism, and acne in the intervention group significantly improved after the research intervention compared to the baseline point of the study (*P* < 0.05). However, in the control group, the mean scores difference in health-related quality of life and its domains, including emotional disturbance, weight, infertility, menstrual, hirsutism, and acne at the baseline point of the study compared to after the intervention, were not statistically significant (*P* > 0.05) (Table 3).

## 4. Discussion

To the best of our knowledge, it seems the present study is the first studying the effect of acupressure on the health-related quality of life of patients with PCOS. In the discussion, since no study similar to the present study was found, the results of this study were compared to studies that use similar mechanisms of acupressure, such as acupuncture and auriculotherapy.

The results indicated that in the intervention group, the mean total testosterone decreased compared to the control group, indicating the effectiveness of the intervention in the present study. In the study by Lim et al., a significant decrease in total testosterone was reported in the intervention group under acupuncture [20]. Moreover, in the study by Johansson et al. 2013, the frequency of ovulation increased in the acupuncture group compared to the control group and the testosterone level decreased. Auriculotherapy, electroacupuncture, and acupressure improve the hormonal balance by modulating the hypothalamic-pituitary-ovarian axis. It leads to a reduction in testosterone levels [30]. Similar to the present study, in the study of Shi et al. 2009, the results showed that acupuncture combined with Chinese herbs has a better therapeutic effect than using only Chinese herbs in patients with PCOS and reduces total testosterone [31]. Although the present study investigates the effect of acupressure on the improvement of total testosterone, since the points used in acupressure and acupuncture are similar and these two have similar effects, the results of the above studies are consistent with the results of this study. Moreover, decreasing testosterone reduces endocrine disorders and can help alleviate PCOS disorders.

The results of the present study indicated the effect of acupressure on the clinical symptoms of acne, hirsutism, and alopecia. Consistent with the results of the present study, Jedel et al. displayed the effectiveness of electroacupuncture in reducing the symptoms of hyperandrogenism, acne, and menstrual disturbance [32].

This study indicates the positive effects of acupressure on health-related quality of life and domains, including hirsutism, acne, menstrual disturbance, weight, emotional disturbance, and infertility in patients with PCO. Stener-Victorin et al., in line with this study, indicated that acupuncture is effective in the health-related quality of life among patients with PCOS [33]. Furthermore, in a study by Witt et al., electroacupuncture significantly improved patients' quality of life with dysmenorrhea [34]. Due to the similarity of the mechanism of action of acupuncture and acupressure, acupressure had improved the quality of life of patients with PCOS in the present study.

The results of the present study indicate that in the acupressure intervention group, menstruation improved, and weight likewise was reduced. According to the results of the present study, the findings of the study of Lim et al. revealed that acupuncture significantly improved menstruation [20]. Correspondingly, in a study by Witt et al. and Qu et al., electroacupuncture significantly improved menstrual pain intensity [34] and the menstrual cycle, respectively [35]. Chen et al. as well examined the therapeutic effect of acupressure on Sp6, Gb32, and Liv3 points and showed that acupressure has long-term effects and reduces menstrual pain and subsequent low back pain [36]. The similarity of the mentioned study with the present study is due to the use of pressure points Sp6 and Liv3 and the effect of acupressure on relieving blood stasis and consequently, relieving dysmenorrhea and reducing menstrual problems. [35]. Nevertheless, according to the study by Stener-Victorin et al., electropuncture intervention did not cause weight loss in patients with PCOS [37]. Perhaps, the difference between the results of these two studies was due to the smaller number of samples, less frequency of intervention, and shorter follow-up time in this study than in the present study. Acupressure of the joints may increase insulin sensitivity in obese or overweight women with PCOS. The guideline recommends the clinical practice of exercise and weight loss as treatments for PCOS.

Furthermore, emotional problems were reduced in the present study, as the study by Stener-Victorin et al. indicated the effect of acupuncture on reducing anxiety and depression. [33] Acupressure can improve the regulation of cortisol secretion and ultimately reduce anxiety by increasing the production of serotonin and endorphins [38].

Thus, acupressure and improving endocrine function can help regulate hormones and reduce mental disorders in patients with PCOS. Correspondingly, Valiani et al. revealed that auriculotherapy reduces stress and improves fertility treatment [39].

One of the limitations of the research was the short duration of follow up. The questionnaires were answered based on self-declaration in which responding factors maybe distort responses.

One of the strengths of the present study is enough sample size, which increases the power of statistical analysis. Moreover, a specific questionnaire related to the quality of life of patients with PCOS was used. Pressure on sham points was used in the control group. All interventions were performed by one researcher.

## 5. Conclusions

The present study indicated the effectiveness of acupressure in reducing total testosterone. The results revealed the improvement of symptoms and health-related quality of life in patients with PCOS.

Since acupressure is one of the nonpharmacological complementary methods, it is non-invasive, relatively cheap, and has no side effects, and can be applied even by the individual. According to the results of this study, acupressure, along with other standard treatments, can be used to promote the health-related quality of life. However, further studies are required to confirm the results of the present study.

## Figures and Tables

**Figure 1:** Location of points; red: acupressure point; green: placebo point. (a) Liv3 and placebo points, (b) SP6 and placebo points, (c) SP10 and placebo points, and (d) REN 3, REN 4, and placebo.

**Figure 2:** Flow diagram of patient's enrolment and study progress.

**Table 1:** Comparison of demographic characteristics between the two groups at baseline.

Variables		Control *N* = 48	Intervention *N* = 48	Total *N* = 96	*P* value
Ethnicity *N* (%)	Fars	18 (37.4)	24 (50)	42 (43.8)	0.32^*∗*^
	Lor	22 (45.8)	20 (41, 7)	42 (43.8)	
	Turkish	8 (16.7)	4 (8.3)	12 (12.4)	

Education *N* (%)	Elementary	18 (37.2)	9 (18.8)	27 (28.1)	0.1^*∗*^
	High school	16 (33.3)	24 (50)	40 (41.7)	
	Diploma and higher	14 (29.2)	15 (31.2)	29 (30.2)	

Employment *N* (%)	Employer	13 (27.1)	11 (22.9)	24 (25)	0.64^*∗*^
	Housewife	35 (72.9)	37 (77.1)	72 (75)	

Menstruation problems *N* (%)	Regular	15 (3.31)	12 (25)	27 (28.1)	0.74^*∗*^
	Irregular	14 (29.2)	19 (39.6)	33 (34.4)	
	Less than 21 days	15 (31.3)	14 (29.2)	29 (30.2)	
	More than 35 days	4 (8, 2)	3 (6, 2)	7 (7.3)	

Infertility *N* (%)	Primary	32 (66.7)	28 (58.3)	60 (62.5)	0.4^*∗*^
	Secondary	16 (33.3)	20 (41.7)	36 (37.5)	

Number of children *N* (%)	1	18 (37.5)	14 (29.2)	32 (33.3)	0.47^&^
	2	20 (41.7)	19 (39.6)	39 (40.7)	
	3 and more	10 (20.8)	15 (31.2)	25 (26)	

Age (years) (mean ± SD)		32.8 ± 2.7	32.6 ± 3.4		0.74^∗∗^

BMI (mean ± SD)		26.2 ± 2.1	26.8 ± 2.2		0.18^∗∗^

Infertile (years) (mean ± SD)		3.1 ± 1.3	2.9 ± 1.2		0.4^∗∗^

^*∗*^Based on independent *t*-test, ^∗∗^chi-square test, *N* (%) = number (percent).

**Table 2:** Comparison of clinical symptoms, total testosterone, and HRQOL of women with polycystic ovarian syndrome between study groups.

Variables		Time	Mean ± dtandarddeviation		MeanDifference	Independent*t*-test	
			Intervention	Control		t	Sig. (2-tailed)
Clinical symptoms	Acne	Before	7.3 ± 2.9	6.7 ± 2.1	0.563	1.10	0.28
		After	5.3 ± 1.9	6.4 ± 2.1	−1.083	−2.64	0.01
	Hirsutism	Before	8.3 ± 3.1	8.1 ± 1.9	0.229	0.44	0.66
		After	5.8 ± 1.5	7.6 ± 2.4	−1.854	−4.50	0.001
	Alopecia	Before	1.7 ± 0.7	1.6 ± 0.7	0.125	0.92	0.36
		After	1.3 ± 0.5	1.6 ± 0.7	−0.313	−2.58	0.01

Total testosterone (Ng/DL)		Before	4.3 ± 1.1	4.1 ± 0.8	0.250	1.28	0.20
		After	2.7 ± 0.6	3.8 ± 1.2	−1.104	−5.72	0.001

HRQOL scores		Before	107.5 ± 5.8	107.1 ± 5.6	0.396	0.34	0.74
		After	120.6 ± 5.5	108.3 ± 4.4	12.292	12.16	0.001

Domains of HRQOL	Emotionaldisturbance	Before	24.3 ± 3.4	25.2 ± 2.8	−0.813	−1.29	0.20
		After	26.3 ± 2.2	24.3 ± 2.8	2.000	3.91	0.001
	Weight	Before	21.5 ± 2.2	21.3 ± 2.1	0.188	0.44	0.66
		After	22.7 ± 2.3	21.1 ± 2.1	1.542	3.46	0.001
	Infertility	Before	10.4 ± 1.4	10.2 ± 1.7	0.250	0.78	0.44
		After	12.2 ± 1.8	10.8 ± 1.7	1.417	4.04	0.001
	Menstrualdisturbance	Before	18.2 ± 2.1	17.5 ± 2.8	0.771	1.56	0.12
		After	21.4 ± 3.3	18.2 ± 2.5	3.250	5.51	0.001
	Hirsutism	Before	18.5 ± 2.6	18.5 ± 3.3	−0.042	−0.07	0.95
		After	21.6 ± 2.7	19.3 ± 3.1	2.313	3.93	0.001
	Acne	Before	14.5 ± 2.1	14.5 ± 2.2	0.042	0.10	0.93
		After	16.4 ± 2.3	14.7 ± 2.1	1.729	3.82	0.001

^*∗*^Based on independent *t*-test., M ± SD = mean ± standard deviation.

**Table 3:** Comparison of clinical symptoms, total testosterone, and HRQOL of women with polycystic ovarian syndrome within study groups.

Variables			Time	Before	After	*P* value^*∗*^
				M ± SD	M ± SD	
Clinical symptoms		Acne	Intervention	7.3 ± 2.9	5.3 ± 1.9	0.001
			Control	6.7 ± 2.1	6.4 ± 2.1	0.32
		Hirsutism	Intervention	8.3 ± 3	5.8 ± 1.5	0.001
			Control	8 ± 1.9	7.6 ± 2.4	0.36
		Alopecia	Intervention	1.7 ± 0.7	1.3 ± 0.5	0.001
			Control	1.6 ± 0.7	1.6 ± 0.7	0.88

Total testosterone (Ng/DL)			Intervention	4.3 ± 1.1	2.7 ± 0.6	0.001
			Control	4.1 ± 0.8	3.8 ± 1,	0.14

HRQOL			Intervention	107.5 ± 5.8	120.6 ± 5.5	0.001
			Control	107.1 ± 5.6	108.3 ± 4.4	0.27

Domains of HRQOL	Emotional disturbance		Intervention	24.3 ± 3.4	26.3 ± 2.2	0.002
			Control	25.2 ± 2.8	24.3 ± 2.8	0.15
	Weight		Intervention	21.5 ± 2.2	22.7 ± 2.3	0.02
			Control	21.3 ± 2.1	21.1 ± 2.1	0.68
	Infertility		Intervention	10.4 ± 1.4	12.2 ± 1.8	0.001
			Control	10.2 ± 1.7	10.8 ± 1.7	0.07
	Menstrual disturbance		Intervention	18.2 ± 2.1	21.4 ± 3.3	0.001
			Control	17.5 ± 2.8	18.2 ± 2.5	0.17
	Hirsutism		Intervention	18.5 ± 2.6	21.6 ± 2.7	0.001
			Control	18.5 ± 3.3	19.3 ± 3.1	0.18
	Acne		Intervention	14.5 ± 2.1	16.4 ± 2.3	0.001
			Control	14.5 ± 2.2	14.7 ± 2.1	0.68

^*∗*^Based on pair *t*-test, M ± SD = mean ± standard deviation.

## Data Availability

The data used to support the findings of this study are available upon request from the first author.
